RETRACTED

# Role of miR-181b/Notch1 Axis in circ_TNPO1 Promotion of Proliferation and Migration of Atherosclerotic Vascular Smooth Muscle Cells

**DOI:** 10.1155/2022/4086935

**Published:** 2022-03-27

**Authors:** Mingxiang Chen, Fuping Li, Qilong Jiang, WeiMin Zhang, Zhiping Li, Wenshuai Tang

**Affiliations:** Department of Cardiovascular Surgery, The Third Affiliated Hospital Of Chongqing Medical University, Chongqing, China

## Abstract

**Background:**

The role and expression level change in circ_TNPO1 (hsa_circ_0072951) in atherosclerosis (AS) and VSMC dysfunction remain unknown. In this study, we try to explore the effects of circ_TNPO1 on oxidized low-density lipoprotein (ox-LDL)-induced human vascular smooth muscle cell (VSMC) excessive proliferation and migration, and the potential molecular mechanism.

**Methods:**

Quantitative real-time polymerase chain reaction (RT-qPCR) and western blot experiment were used to detect the serum samples from AS patients and healthy controls. CCK-8, Transwell, and the dual-luciferase reporter gene assay were used to detect the cell biology.

**Results:**

In human AS serum and ox-LDL-induced VSMCs, circ_TNPO1 was increased, whereas miR-181b was decreased. Silencing circ_TNPO1 inhibited proliferation and migration activity and reduced protein expression of PCNA, Ki-67, MMP2, and E-cadherin and promoted N-cadherin protein expression in ox-LDL induced VSMCs. Remarkably, miR-181b knockdown or Notch1 overexpression could efficiently offset the proliferation and migration inhibiting effect of circ_TNPO1 knockdown in ox-LDL-induced VSMCs. Furthermore, a molecular mechanism study pointed out that circ_TNPO1 and Notch1 are direct-acting targets of miR-181b.

**Conclusions:**

In conclusion, our study indicated that circ_TNPO1 promotes the proliferation and migration progression of VSMCs in atherosclerosis through the miR-181b/Notch1 axis.

## 1. Introduction

In recent years, the incidence of atherosclerosis (AS) had an increasing trend worldwide year by year [1]. Atherosclerotic plaque rupture following a lead to acute thrombosis is an important cause of cerebral infarction and acute myocardial infarction [2]. Numerous studies have pointed out that the proliferation, invasion, and migration of VSMCs originating from the middle arterial layer are playing a significant role in the pathological processes of atherosclerotic plaque formation [3, 4]. In normal arteries, VSMCs regulate the contraction of arteries and modulate the synthesis of the extracellular matrix. In AS, VSMCs migrate from the media layer to the intima and switch from a “contractile” phenotype to an activated “synthetic” phenotype. Synthetic VSMCs generally demonstrate enhanced viability in cell proliferation and migration and could exacerbate inflammatory response and intimal calcification, ultimately promoting the process of atherosclerosis [5, 6]. The abnormal proliferation and migration of VSMCs are critical events of atherosclerosis. Thus, it is extremely important to investigate the molecular mechanisms of excessive proliferation and migration of VSMCs to treat and prevent AS.

RETRACTED

Circular RNAs (circRNAs) are a class of noncoding RNAs characterized by covalently linked 5' and 3′ ends with a closed circular structure. Current studies point out that some upstream regulators of circRNA biogenesis or stability have been studied already before the rediscovery of circRNAs in the context of AS [7, 8]. circRNA plays an indirect role in regulating mRNA translation. mRNA translation contains miRNA response elements and acts as a miRNA sponge to inhibit miRNA-mediated repression of target mRNA， thus regulating the pathologic process of AS [9]. circRNAs are the latest focus of atherosclerotic pathology and are involved in regulating the proliferation and migration process of VSMCs. However, the key circRNAs regulating the proliferation and migration process of VSMCs cells and their precise mechanism remain unclear. circ_TNPO1 (hsa_circ_0072951) is located on chromosome 5. No research has yet been reported on the regulatory effect of circ_TNPO1 in AS and the dysfunction of VSMCs. In this study, we investigated the expression level variation of circ_TNPO1 in the serum of AS patients and correlations between circ_TNPO1 and VSMC dysfunction.

MicroRNA (miRNA) is an important post-transcriptional level regulator, which can bind to the 3′ untranslated region (3′-UTR) of mRNA, leading to translation inhibition or degradation of mRNA. Recent studies have pointed out that the decreased expression level of miR-181b may be an important cause of AS plaque formation and vascular endothelial injury [10, 11]. The reason for reduced expression levels of miR-181b in AS is not known. Prior studies have suggested that miR-181b exerted these biological effects by directly repressing Notch1. The Notch1 proteins are evolutionarily conserved transmembrane receptor proteins that are widely distributed in a variety of tissue [12]. Recent research indicated that Notch1 signaling is significantly activated in AS plaques, and overexpression of Notch1 can promote proliferation, migration, survival, and extracellular matrix synthesis of VSMCs [13–15].

In this study, we investigated the expression level variation of circ_TNPO1 in the serum of AS patients and correlations between circ_TNPO1 and VSMCs dysfunction and to verify whether it exerts its biological effects by targeting the miR-181b/Notch1 axis.

RETRACTED

## 2. Methods

### 2.1. Serum Samples

The 37 patients with AS were included from the clinic and inpatient department of The Third Affiliated Hospital of Chongqing Medical University between June 2019 and June 2020. Written informed consent was obtained from all patients before collecting their serum samples. Additionally, 40 serum samples from healthy individuals were collected during the same period as the control group. For all patients, 5 ml of morning fasting venous blood was collected and centrifuged at 4,000 r/min for 10 min, and the separated serum was stored in a refrigerator at -80°C.

### 2.2. circRNA Sequence

circRNA sequences were conducted as in the literature [10]. The sequencing experiments were performed by Shanghai Yuansong Biotechnology Co., Ltd.

### 2.3. RT-qPCR Experiment

Serum samples from AS patients and healthy controls were collected. Then, total RNA was extracted from serum samples using TRIzol reagent (TRIzol reagent, Sigma-Aldrich, St. Louis, Missouri). Total RNA was precipitated with isopropanol and then dissolved with DEPC-H2 (General Biotech). cDNA was synthesized by M-MLV-reverse transferase using an RT-PCR kit (Promega) according to the kit instructions. qPCR amplification was performed using ABI 7300 real-time PCR system (Applied Biosystems) using 2X Power SYBR-Green PCR Master Mix (Applied Biosystems) according to the kit instructions (Table 1). The relative expression of mRNA was determined by the relative standard curve method (2^−ΔΔCt^) using GAPDH as an internal reference.

### 2.4. Western Blot Experiment

The protein samples were prepared and stored at -80°C. After denaturation, the proteins were separated by 10% SDS-PAGE gel electrophoresis. Then, the proteins were transferred to the PVDF membrane (Millipore, USA) by the wet transfer method. Subsequently, PVDF membrane was incubated with 5% skimmed milk powder for 2 h, washed three times with TBST, incubated overnight at 4°C with primary antibody, incubated for 1h at room temperature with secondary antibody, washed four times with TBST, and detected by Odyssey two-color infrared fluorescence imaging system (LI-COR Company, USA). The immunoreactive bands on the membrane were detected using the Odyssey two-color IR imaging system.

### 2.5. Cell Culture

Human VSMCs (ScienCell, no. 6,110) were cultured in a DMEM medium (GIBCO, USA) containing 10% fetal bovine serum (GIBCO, USA) at 37°C in a humidified incubator with 5% CO_2_. When cell density grew to 80%, the supernatant was discarded and the digestion proceeded with 0.25% trypsin-EDTA for cell passages. The ox-LDL-induced AS model was conducted as shown in the literature and is briefly described here as follows. VSMCs of the experimental group were treated with 30, 60, 90, or 120 *μ*g/mL ox-LDL for 24 h, while VSMCs of the control group with the same volume of solution without ox-LDL.

RETRACTED

### 2.6. CCK-8 Assay

After transfection, cells in each group were cultured for 48 h, then, 10 *μ*L CCK-8 reagent (Dojindo, Japan) was added into each well, and the absorbance at 570 nm was measured by microplate reader after 2-h incubation.

### 2.7. Transwell Assay

After transfection, cells in each group were collected. Then, 1 × 10^5^ cells suspended in 200 *μ*l serum-free DMEM media were inoculated into the upper layer of Transwell (Corning, USA) for 24 h. After the VSMCs had been cultured for 24 h, the upper layer of cells was gently wiped off with a cotton swab, subsequently, were washed with PBS, fixed with 4% paraformaldehyde for 30 min, and then stained with 0.1% crystal violet (Nakaraitesk, Kyoto, Japan) for 10 min. Finally, 3 fields of view were randomly selected under an inverted microscope for photographing and counting. The experiment was repeated 3 times.

### 2.8. Dual-Luciferase Reporter Gene Assay

The wild sequence or mutant sequence of Notch1 (3′-UTR) and circ_TNPO1 containing miR-181b binding site was cloned into the psiCHECK plasmid to construct dual-luciferase reporter plasmids. Afterward, miR-181b mimic or miR-NC (GenePharma, China) was cotransfected with WT or MUT plasmids into VSMCs, respectively. Cells were collected 48 h after transfection, and luciferase activity was detected using a dual-luciferase reporter gene assay kit (Promega, USA).

### 2.9. Cell Transfection

The VSMCs were seeded in a T-25 cm^2^ flask and related si-RNAs, and pcDNA plasmid was transfected with Lipofectamine 3000 (Invitrogen, USA) after reaching a density of 50%–60% confluence. These si-RNA and pcDNA plasmids included si-circ_TNPO1, miR-181b mimic, miR-181b inhibitor, pcDNA plasmid (Notch1), and the negative controls (si-NC, miR-NC, and empty pcDNA plasmid). The sequence of oligonucleotides is depicted below as follows: si-circ_TNPO1, 5′-AAGTTGTTTAACTATAGTCCTTC-3′; si-NC, 5′-GCAAGCTGACCCTGAAGTT-3′; miR-181b mimic, 5′-AACAUUCAUUGCUGUCGGUGGGU-3′; miR-181b inhibitor, 5′−ACCCACCGACAGCAAUGAAUGUU−3′; miR-NC, 5′-GCUUCAUACGUGGACUAAUCU-3′; miR-inhibitor NC, 5′-CAGCACUCAUGUAUGGUACGG-3′.

### 2.10. Statistical Analysis

SPSS 17.0 statistical software was used for statistical analysis. Quantitative data were expressed as mean ± standard deviation (mean ± SD). The *t*-test was used for comparison between two groups, and *P* < 0.05 was considered a statistically significant difference.

## 3. Results

### 3.1. Expression Level of circ_TNPO1 Was Increased in AS Patients' Serum and Ox-LDL-Treated VSMCs

By circular RNA sequence method, overall 33 circRNAs were significantly differentially expressed with the screening criteria: *P* < 0.05, fold change>2.0, or fold change < −2.0. Among them, circ_TNPO1 was the most significantly upregulated circRNA, as shown in Figure 1(a). Subsequently, an RT-qPCR assay was performed to validate the reliability of the results of the circRNA sequencing experiment. Consistent with the result of circRNA sequence, RT-qPCR assay pointed out that the expression of circ_TNPO1 was significantly increased in the serum of AS patients compared with the control group, as shown in Figure 1(b).

RETRACTED

A large number of research indicated that ox-LDL is a potential inducer of VSMC dysfunction in AS. Thus, we treated VSMCs with different doses of ox-LDL. These results indicated that, *in vitro* level, ox-LDL promoted the expression of circ_TNPO1 in a dose-dependent manner. In summary, our study suggests that circ_TNPO1 expression is significantly increased in the serum of AS patients and ox-LDL-treated VSMC and may be a key pathogenic determinant of AS.

### 3.2. The Knockdown of circ_TNPO1 Inhibited Proliferation and Migration Progression of Ox-LDL-Induced VSMCs

To investigate the functional role of circ_TNPO1 in ox-LDL-induced proliferation and migration of VSMCs, we applied si-RNA transfection to artificially knockdown circ_TNPO1 expression level in VSMCs. RT-qPCR identified that the expression level of circ_TNPO1 was significantly reduced in VSMCs transfected with si-circ_TNPO1, as shown in Figure 2(a). Subsequently, loss function experiments were performed in ox-LDL-treated VSMCs. CCK-8 assay revealed that the si-circ_TNPO1 treatment dramatically attenuates proliferation activity of ox-LDL-treated VSMCs at 24 h, as shown in Figure 2(b). Moreover, si-circ_TNPO1 treatment dramatically reduced Ki-67 and PCNA protein expression levels in ox-LDL-treated VSMCs, which was consistent with the results of the CCK-8 assay, as shown in Figure 2(d). Transwell assay indicated that the number of migrating VSMCs in the si-circ_TNPO1-treated group was significantly lower compared with the si-NC-treated group, as shown in Figure 2(c). Consistent with the results of the Transwell assay, Western blot analysis also indicated that si-circ_TNPO1 treatment dramatically reduced MMP2 and N-cadherin protein expression level, while the expression levels of E-cadherin proteins were significantly promoted, as shown in Figure 2(d). In summary, our study suggests that knockdown of circ_TNPO1 could significantly inhibit ox-LDL-induced proliferation and migration of VSMCs.

### 3.3. miR-181b Directly Interacted with circ_TNPO1 in VSMCs

Previous studies have shown that the knockdown of circ_TNPO1 inhibited proliferation and migration progression of ox-LDL-induced VSMCs. To further explore the molecular mechanism of circ_TNPO1, we predicted the potential targets of circ_TNPO1 based on the TargetScan database. The results showed that circ_TNPO1 has a miR-181b binding site, as shown in Figure 3(a). Pearson's correlation coefficient analysis showed that circ_TNPO1 was negatively correlated with miR-181b, as shown in Figure 3(b). RT-qPCR assay pointed out that the expression of miR-181b was significantly decreased in the serum of AS patients compared with the control group, as shown in Figure 3(c).

RETRACTED

Finally, a dual-luciferase reporter assay was used to verify the direct interaction between circ_TNPO1 and miR-181b. The results showed that miR-181b mimic cotransfected with WT plasmid was able to significantly reduce luciferase activity in VSMCs. However, miR-181b mimics cotransfected with MUT plasmid did not reduce luciferase activity in VSMCs, as shown in Figure 3(d). These outcomes illuminated that circ_TNPO1 may exert its biological function by targeting miR-181b.

### 3.4. The Blockage of miR-181b Counteracted Proliferation and Migration Suppressing Effects of circ_TNPO1 Knockdown in Ox-LDL-Induced VSMCs

Our studies have shown that miR-181b is a direct target of circ_TNPO1, and si-circ_TNPO1 treatment dramatically promotes the expression level of miR-181b in VSMCs, yet whether circ_TNPO1 exerts its biological effects by targeting miR-181b is not directly verified. To further prove whether the proliferation and migration suppressing effects of circ_TNPO1 knockdown rely on overexpression of miR-181b, we carried out a rescue experiment.

RT-qPCR assay indicated that miR-181b inhibitor transfection can significantly suppress the expression level of miR-181b， as shown in Figure 4(a). Rescue experiment indicated that miR-181b inhibitor transfection can significantly facilitate the activity of proliferation and migration in VSMCs with circ_TNPO1 depletion under ox-LDL stress， as shown in Figures 4(b) and 4(c). Subsequently, consistent with the results of CCK-8 assay and Transwell assay, Western blot analysis also indicated that miR-181b inhibitor transfection can significantly promote protein expression level of Ki-67, PCNA, MMP2, and E-cadherin while inhibiting protein expression level of N-cadherin in VSMCs with circ_TNPO1 depletion under ox-LDL stress, as shown in Figure 4(d). These outcomes indicated that the blockage of miR-181b counteracted proliferation and migration suppressing effects of circ_TNPO1 knockdown in ox-LDL-induced VSMCs.

RETRACTED

### 3.5. miR-181b Directly Interacted with Notch1 in VSMCs

It has been shown that miR-181b has a direct interaction with Notch1 in other cell lines. In this study, we predicted the potential targets of miR-181b based on the TargetScan database. The results showed that miR-181b had binding sites with Notch1, as shown in Figure 5(a). Pearson's correlation coefficient analysis showed that miR-181b was negatively correlated with Notch1, while Notch1 was positively correlated with circ_TNPO1, as shown in Figure 5(b). Moreover, RT-qPCR assay indicated that the expression level of Notch1 was dramatically increased in ox-LDL-induced VSMCs and VSMCs transfected with si-circ_TNPO1, as shown in Figure 5(c). Subsequently, RT-qPCR assay indicated that miR-181b inhibitor can dramatically promote mRNA and protein expression levels of Notch1. All these findings suggest that Notch1 may be a direct target of miR-181b. Finally, a dual-luciferase reporter assay was used to verify the direct interaction between Notch1 and miR-181b. Dual-luciferase reporter assay showed that miR-181b mimic cotransfected with Notch1 WT plasmid was able to significantly reduce luciferase activity in VSMCs. However, miR-181b mimic cotransfected with Notch1 MUT plasmid did not inhibit luciferase activity, as shown in Figure 5(d). These outcomes illuminated that miR-181b directly interacted with Notch1 in VSMCs.

### 3.6. Overexpression of Notch1 Counteracted Inhibition Effects of Proliferation and Migration of circ_TNPO1 Knockdown in Ox-LDL-Induced Human VSMCs

Notch1 has been well demonstrated to promote cell proliferation and migration in a variety of cell lines. Previous studies have well demonstrated that circ_TNPO1 may promote Notch1 expression by targeting miR-181b in ox-LDL-treated VSMCs; however, whether circ_TNPO1 exerts its pro-proliferative and migratory effects on VSMCs through overexpression of Notch1 is unclear. The overexpression experiment indicated that Notch1 overexpression can restore the content of Notch1 in VSMCs transfected with si-circ_TNPO1, as shown in Figures 6(a) and 6(b). In addition, CCK-8 and Transwell assay indicated that restoring Notch1 expression also can augment the activity of proliferation and migration in VSMCs with circ_TNPO1 depletion under ox-LDL stress, as shown in Figures 6(c) and 6(d). Subsequently, Western blot analysis also indicated that si-circ_TNPO1 lowered protein expression of Ki-67, PCNA, MMP2, and E-cadherin and enhanced protein expression of N-cadherin in ox-LDL-induced VSMCs, which was rescued by Notch1 overexpression plasmid, as shown in Figure 6(e). These outcomes indicated that overexpression of Notch1 counteracted inhibition effects of proliferation and migration of circ_TNPO1 knockdown in ox-LDL-induced human VSMCs.

RETRACTED

## 4. Discussion

circRNAs are endogenous noncoding RNAs, which are a hot topic of current research. Currently, with the continuous progress of detection technology, more and more circRNAs are discovered and their mechanisms of action are gradually revealed. A large number of studies have shown that circRNAs can play an important role in the development and progression of VSMC dysfunction and AS by acting as molecular sponges for miRNAs and exerting ceRNA mechanisms to indirectly regulate the expression of target genes. For example, Ding [16] et al. showed that in ox-LDL-induced VSMCs, circ_0010283 promoted the proliferation and migration of VSMCs through the miR-370-3p/HMGB1 axis. Wang et al. [17] showed that circ_CHFR was able to promote the proliferation, invasion, and migration of VSMCs through the miR-149-5p/NRP2 axis under the induction of PDGF-BB. VSMCs are the major cellular components of arteries, a special class of multiphenotypic and multifunctional cellular taxa. When the blood vessels are stimulated by pathological factors, multiple signaling pathways on VSMCs are activated and the number of “synthetic” phenotypes of VSMCs gradually increases. While synthetic VSMCs have the functions of secretion, migration, and proliferation, the excessive proliferation and migration of VSMCs are the pathophysiological basis of atherosclerosis and vascular stenosis diseases [18, 19].

circRNAs can be used as early predictors of AS development and provide more effective biomarkers for the diagnosis and treatment of AS [20]. However, the expression of profile regulatory mechanisms of most circRNAs in the pathological process of AS remains poorly known. No study has been conducted to investigate the effect of circ_TNPO1 on the proliferation and migration of VSMCs and potential mechanisms. In this study, circRNA sequencing technology was used to detect the differentially expressed circRNAs between the AS patients' serum and healthy controls, and from them, we found that circ_TNPO1 expression levels were significantly increased in the serum of AS patients. Subsequent RT-qPCR results further indicated that circ_TNPO1 expression was significantly increased in ox-LDL-treated VSMCs and the serum of AS patients. Subsequently, the function studies indicated that knockdown of circ_TNPO1 significantly inhibited proliferation and migration progression of ox-LDL-induced VSMCs. Subsequently, a molecular mechanism study indicated that, under ox-LDL stress, circ_TNPO1 could indirectly regulate the expression level of Notch1 by targeting miR-181, thus promoting the proliferation and migration progression of VSMCs.

RETRACTED

In this study, the results of the RT-qPCR assay pointed out that expression levels of miR-181b were significantly downregulated in the serum of AS patients. Consistent with our findings, the results of Li and Cao and Zhong et al. [21, 22] pointed out that expression levels of miR-181b were significantly reduced in the serum of patients with atherosclerosis. In addition, our study also demonstrated that miR-181b expression levels were also significantly downregulated in ox-LDL-treated VSMCs, which is consistent with the previous findings [23].

Subsequently, the dual-luciferase reporter assay indicated that miR-181b directly interacted with circ_TNPO1 in VSMCs. Regarding the effect of miR-181b on the proliferation and migration of VSMCs, our results pointed out that miR-181b knockdown significantly promoted abilities of proliferation and migration of ox-LDL induced VSMCs transfected with si-circ_TNPO1 and promoted Ki67, PCNA, MMP2, and E-cadherin protein expressions. Consistent with our findings, the results of Ghasempour et al. [23] indicated that miR-181b was able to inhibit the proliferation and migration of VSMCs by regulating the *β*-ARR2/p-ERK1/2 signaling pathway. Also, the results of Ghasempour et al. [24] indicated that miR-181b could inhibit the proliferation and migration of VSMCs by targeting HCK, and in addition, the results of Zhong et al. [21] indicated that miR-181b could inhibit cell proliferation by targeting STAT3 in an ox-LDL-induced AS cell model and inhibiting cell cycle to promote apoptosis. Taken together, miR-181b may provide a new therapeutic target for alleviating the disease process of AS.

In our study, further molecular mechanism study indicated that miR-181b directly binds to the 3′-UTR of Notch1 mRNA and thus inhibits Notch1 expression on mRNA and protein level in VSMCs. Currently, the interactive relationship between miR-181b and Notch1 has been widely reported in a variety of cell lines. In addition, our results showed that Notch1 expression levels were increased in serum samples from AS patients and showed a trend toward a positive association with circ_TNPO1 expression level and a negative association with miR-181b expression level. Our results align with the findings from previous studies. For instance, Bassani et al. [25] pointed out that miR-181b was able to target Notch1 and inhibit Notch1 expression in human NK cells. Moreover, An et al. and Sun et al. [10, 11] also pointed out that the presence of a direct interact relationship between miR-181b and Notch1 and miR-181b/Notch1 axis plays a significant role in the pathogenesis of AS. Subsequently, function studies indicated that the overexpression of Notch1 counteracted the knockdown of circ_TNPO1 induced inhibitory effects of proliferation and migration of VSMCs under ox-LDL stress. Notch1 plays an important regulatory role in the proliferation and migration of VSMCs, and its possible mechanisms include the CBF-1/RBP-J*κ*-dependent pathway and the non-CSL-dependent pathway [26]. Consistent with our findings, Chen et al. [27] showed that miR-34a was able to inhibit VSMCs cell proliferation and migration by targeting the 3′-UTR of Notch1.

RETRACTED

Our study also indicated that si-circ_TNPO1 lowered protein expression of Ki-67, PCNA, MMP2, and E-cadherin and enhanced protein expression of N-cadherin in ox-LDL-induced VSMCs， which was rescued by Notch1 overexpression plasmid. Ki-67 and PCNA are the most common markers reflecting cell proliferation. MMP2 and E-cadherin are molecular markers of cell migration. E-cadherin is a transmembrane glycoprotein that binds normal and polarized epithelial cells together at adhesion junctions, thereby inhibiting abnormal cell proliferation and migration. MMP2 is a protein with type IV collagen degradation properties that has a biological function in promoting cell migration. The correlation between Notch1, MMP2, and E-cadherin protein expressions has been investigated. For example, Fujiki et al. [26] noted that the application of si-RNA to inhibit Notch1 expression significantly promoted E-cadherin protein expression in the BEAS-2B cell line. In addition, Wang et al. [27] noted that inhibition of suppression of Notch1 expression in skin cancer cell lines was able to significantly promote E-cadherin protein expression. Meanwhile, Zou et al. [28] pointed out that promoting Notch1 activation promotes MMP2 protein expression levels in Jurkat and Sup-T1 cell lines. However, there are also limitations of this study. There are no animal experiments in this study, which made this study not so scientific.

Taken together, our study shows that circ_TNPO1 knockdown can inhibit the abnormal proliferation and migration of ox-LDL-induced VSMCs through the miR-181b/Notch1 axis. The results of this study suggest that circ_TNPO1, miR-181b, and Notch1 may be potential therapeutic targets in AS [29, 30].

## Figures and Tables

**Figure 1:** circ_TNPO1 expression was significantly increased in serum of AS patients and ox-LDL-treated VSMCs. (a) A heat map with hierarchical clustering of 33 differentially expressed circRNAs between AS serum and healthy controls serum. (b) Relative circ_TNPO1 expression levels in AS sample and control sample were determined by RT-qPCR. (c) The expression level of circ_TNPO1 in VSMCs treated by different doses of ox-LDL was detected by RT-qPCR. ^*∗*^*P* < 0.05.

RETRACTED

**Figure 2:** The knockdown of circ_TNPO1 inhibited proliferation and migration progression of ox-LDL-induced VSMCs. (a) Relative expression levels of circ_TNPO1 were measured in VSMCs transfected with si-circ_TNPO1 or si-NC by RT-qPCR assay. (b) CCK-8 assay monitored proliferation activity of VSMCs after cotreatment with si-circ_TNPO1 or si-NC and ox-LDL. (c) Transwell assay monitored migration activity of VSMCs after cotreatment with si-circ_TNPO1 or si-NC and ox-LDL. (d) Western blot assay detected the protein expression levels of Ki67, PCNA, MMP2, E-cadherin, and N-cadherin in VSMCs after cotreatment with si-circ_TNPO1 or si-NC under ox-LDL stress. ^*∗*^*P* < 0.05.

**Figure 3:** miR-181b directly interacted with circ_TNPO1 in VSMCs. (a) TargetScan database predicts the binding sequence between circ_TNPO1 and miR-181b. (b) Pearson's correlation coefficient determined the correlations between circ_TNPO1 and miR-181b in AS patients' serum. (c) Relative expression levels of miR-181b were measured in AS patients' serum and control healthy serum. (d) Dual-luciferase reporter assay determined the direct interaction of circ_TNPO1 with miR-181b in VSMCs. ^*∗*^*P* < 0.05.

**Figure 4:** The blockage of miR-181b counteracted proliferation and migration suppressing effects of circ_TNPO1 knockdown in ox-LDL-induced VSMCs. (a) Relative expression levels of miR-181b were measured in VSMCs transfected with si-circ_TNPO1 alone, si-NC alone, or together with miR-181b inhibitor or miR-NC. (b) CCK-8 assay monitored proliferation activity of VSMCs transfected with si-circ_TNPO1 alone, si-NC alone, or together with miR-181b inhibitor or miR-NC under ox-LDL stress. (c) Transwell assay detected the migration activity of VSMCs transfected with si-circ_TNPO1 alone, si-NC alone, or together with miR-181b inhibitor or miR-NC under ox-LDL stress. (d) Western blot assay detected the protein expression levels of Ki67, PCNA, MMP2, E-cadherin, and N-cadherin in VSMCs transfected with si-circ_TNPO1 alone, si-NC, or together with miR-181b inhibitor or miR-NC under ox-LDL stress. ^*∗*^*P* < 0.05.

**Figure 5:** miR-181b directly interacted with Notch1 in VSMCs. (a) TargetScan database predicts the binding sequence between Notch1 and miR-181b. (b) Pearson's correlation coefficient determined the correlations between Notch1 and circ_TNPO1 or miR-181b in AS patients' serum. (c) Dual-luciferase reporter assay determined the direct interaction of Notch1 with miR-181b in VSMCs.^*∗*^*P* < 0.05. (d) Effects of miR-181b mimic and miR-181b inhibitor on Notch1 protein expression levels in VSMCs.

**Figure 6:** Overexpression of Notch1 counteracted inhibition effects of proliferation and migration of circ_TNPO1 knockdown in ox-LDL-induced human VSMCs. (a) RT-qPCR assay determined Notch1 mRNA expression level in VSMCs transfected with si-NC, or si-circ_TNPO1, or si-circ_TNPO1 along with pcDNA plasmid or si-circ_TNPO1 along with pcDNA-Notch1 plasmid. (b) The effect of Notch1 overexpression on the proliferative activity of ox-LDL-induced VSMCs transfected with si-circ_TNPO1 was determined by the CCK-8 assay. (c) The effect of Notch1 overexpression on the migrating activity of ox-LDL-induced VSMCs transfected with si-circ_TNPO1 was determined by Transwell assay. (d) The effect of Notch1 overexpression on protein expression of Ki67, PCNA, MMP2, E-cadherin, and N-cadherin in ox-LDL-induced VSMCs transfected with si-circ_TNPO1 was determined by Western blot assay. ^*∗*^*P* < 0.05.

RETRACTED

**Table 1:** The primers of RT-qPCR.

Name	Sequence (5′-3′)
circ_TNPO1	AGCTGCTGAATTTTAAAGAGAGT
	AGGCTCCCTTATAGTCTCCA
miR-181b	ACACTCCAGCTGGGAACATTCATTGCTGTCGG
	TGGTGTCGTGGAGTCG
Notch1	GGTGAACTGCTCTGAGGAGATC
	GGATTGCAGTCGTCCACGTTGA

## Data Availability

The data used to support this study are available from the corresponding author upon request.
